RETRACTED

# Effects of Arteriovenous Thrombolysis Combined with Mechanical Thrombectomy on Efficacy and Neurological Function of Acute Cerebral Infarct Patients

**DOI:** 10.1155/2020/9743075

**Published:** 2020-10-09

**Authors:** Tao Ding, Liwen Tang, Bohong Hu, Junxin Yuan, Xiangdong Li, Jun Wen

**Affiliations:** ^1^Department of Neurology, The First People's Hospital, 818 Renmin East Road, Changde City, Hunan Province, China; ^2^Department of General Surgery, The First People's Hospital, 818 Renmin East Road, Changde City, Hunan Province, China

## Abstract

**Objective:**

To investigate the effects of arteriovenous thrombolysis combined with mechanical thrombectomy on clinical efficacy, neurological function, and the changes of nerve injury markers of acute cerebral infarct (ACI) patients.

**Methods:**

A total of 143 cases with ACI admitted to our hospital from June 2017 to June 2019 were elected as research subjects. Among them, 69 cases of patients who received treatment of arteriovenous thrombolysis were considered as group A, and 74 cases of patients who received treatment of arteriovenous thrombolysis combined with mechanical thrombectomy were considered as group B. NIHSS score, clinical efficacy, vascular recanalization, adverse reactions, hemodynamics, neurological injury indexes, duration of coma, length of hospital stay, and prognosis of patients in the two groups were compared.

**Results:**

After treatment, the NIHSS score of group A was higher than that of group B (*P* < 0.05), the clinical efficacy of group B was better than that of group A, and the incidence of adverse reactions was lower than that of group A (*P* < 0.05). There was no difference in vascular recanalization rate, duration of coma, and prognosis between the two groups (*P* > 0.05). Length of hospital stay, maximum peak velocity after treatment (Vs), and mean flow rate (Vm) of group A were lower than those of group B, while vascular resistance index (RI), pulsatility index (PI), serum glutamic acid (Glu), neuron-specific enolase (NES), and S100*β* protein detected by enzyme-linked immunosorbent assay (ELISA) of group A were higher than those of group B (*P* < 0.05).

**Conclusion:**

Arteriovenous thrombolysis combined with mechanical thrombectomy has a significant effect on ACI, with high safety and quick effect. In addition, it has a stronger effect on improving and protecting the neurological function of patients, which is worth promoting in clinical practice.

## 1. Introduction

Acute cerebral infarction (ACI) refers to brain necrosis caused by sudden dearterialization of the brain. This is usually due to atherosclerosis or thrombosis in the arteries supplying blood to the brain, leading to luminal stenosis or even occlusion, resulting in focal acute insufficient blood supply [1, 2]. ACI is currently an extremely common neurological disease worldwide, with a high incidence in the elderly [3]. According to statistics, the incidence of ACI is as high as 20.6% [4]. In recent years, more studies have shown that the incidence of ACI is on the rise year by year, which may also be closely related to the global aging trend [5, 6]. ACI does great harm to the human body. Patients with ACI are usually accompanied by hemiplegia, facial paralysis, and in severe cases, general paralysis and death [7]. Due to the high incidence and high risk of ACI, clinical efforts have been devoted to exploring how to effectively diagnose and treat ACI. At present, although traditional conventional treatment measures can effectively attenuate the clinical symptoms of patients with cerebral infarction, the prognosis is not ideal, and the recurrence of the disease is extremely common [8]. Therefore, finding an effective treatment method for ACI and improving the prognosis of patients is the focus and difficulty of the current clinical studies.

RETRACTED

In the treatment of ACI, the key is to open occluded large vessels and the emphasis is to timely block blood flow obstruction and restore blood flow recanalization. Thrombolytic therapy is the most commonly used method in clinical practice at present for patients meeting the criteria of thrombolysis [9]. Among them, arteriovenous thrombolysis is the more common solution [10]. In recent years, with the improvement and application of minimally invasive techniques, endovascular mechanical thrombectomy has gradually attracted extensive clinical attention [11]. At present, studies have proved that thrombolysis combined with mechanical thrombectomy can effectively improve the clinical efficacy of ACI patients [12]. In order to further clarify the clinical value of thrombolysis combined with mechanical thrombectomy, this experiment compared the influence of the two treatment methods on the neurological function of ACI patients, observed the changes of glutamic acid (Glu), neuron-specific enolase (NES), and S100*β*, aiming to provide references and guidance for the future clinical selection of treatment methods for ACI.

## 2. Materials and Methods

### 2.1. General Data

A total of 143 cases of patients with ACI admitted to our hospital from June 2017 to June 2019 were selected as research subjects to perform prospective analysis. Among them, 69 cases of patients who received treatment of arteriovenous thrombolysis were considered as group A. And 74 cases of patients who received treatment of arteriovenous thrombolysis combined with mechanical thrombectomy were considered as group B. This study has been approved by the ethical committee of our hospital; all patients above have signed the informed consent.

RETRACTED

### 2.2. Inclusion and Exclusion Criteria

The inclusion criteria were as follows: (1) patients' symptoms complied with the clinical manifestations of cerebral infarction, and the cerebral infarction was diagnosed by CT and MRI plain scan; (2) patients confirmed by CTA examination for intracranial macrovascular embolism; (3) patients' indication conformed to intra-arterial thrombolysis, arteriovenous thrombolysis, and intravascular mechanical thrombectomy; (4) patients with an age of 40-70 years; (5) patients with complete case data; and (6) patients without contraindications for interventional surgery such as coagulation disorders.

The exclusion criteria were as follows: (1) patients complicated with other blood disease or tumors; (2) patients with low treatment compliance; (3) patients with a history of cerebral hemorrhage in 6 months and active hemorrhage in two weeks; (4) patients who received treatment of other antibiotics within 3 months before admission; (5) patients with liver or kidney dysfunction, or patients with organ failure; (6) patients with drug allergies; and (7) patients who died during treatment and were expected to live for no more than one month.

## 3. Methods

### 3.1. Therapies

*Anesthesia scheme*: refer to McEvoy [13], general anesthesia was performed with endotracheal intubation, and induction was performed with etomidate of 0.1 mg/kg, fentanyl of 3 *μ*g/kg, and rocuronium of 0.6 mg/kg. At the same time, remifentanil was intravenously pumped at 0.3 *μ*g/(kg/min) and propofol 3-6 mg/(kg/h). Noradrenaline was supplemented with 0.05 *μ*g/(kg/min) to maintain blood pressure at baseline. After 5 min, endotracheal intubation was established for volume-controlled ventilation, with a tidal volume of 480 mL, frequency of 12 times/min, a suction ratio of 1 : 1.5, and oxygen concentration of 100%. Anesthesia was maintained by intravenous anesthesia, with propofol of 3-4 mg/(kg/h), remifentanil of 0.1-0.2 *μ*g/(kg/min), and rocuronium of 20 mg/h.

*Treatment plan of group A*: a total of one million units of urokinase was dissolved in 100 mL 0.9% sodium chloride solution for intravenous infusion, which was completed within 1 h. After anesthesia, interventional angiography was performed to determine the infarction situation and lesion location, and a microcatheter was taken from the femoral artery through the catheter to the distal end of the thrombus site. Urokinase was pumped at 10,000 U/h and completed within 30 min. After completing withdrawal, the same amount of urokinase (10,000 U/min) was pumped into the thrombus and the proximal thrombus, respectively. The catheter was then removed, and the incision was bandaged.

RETRACTED

*Treatment plan of group B*: the thrombolytic method was the same as above. After angiography, the 6F artery sheath was put in and the guidewire was used to send guiding to the lesion under the angiography. The stent was withdrawn after the angiography, and 30 mL of blood was drawn back to prevent the prolapsed thrombus from flowing back into the artery. When the angiography exhibited that mechanical thrombectomy was successful, the arterial sheath was removed to take out the catheter, and the incision was bandaged. The patients in the two groups received treatment of aspirin (100 mg) and clopidogrel (75 mg) orally for 3 months after surgery.

### 3.2. Detection Methods

Fasting venous blood (5 mL) was extracted from the patients before treatment and 3 d after treatment. It was placed at room temperature for 30 min and then centrifuged for 10 min (400 × g) to obtain the upper serum. Glu in serum was detected by high-performance liquid chromatography (HPLC), NES was detected by electrochemiluminescence, and S100*β* was detected by enzyme-linked immunosorbent assay (ELISA, the kit was purchased from Beijing Future Biotech Co., Ltd., KT-435).

### 3.3. Outcome Measures

*NIHSS score*: Evaluation was performed before treatment and 10 d after treatment. *Clinical efficacy*: After 24 h of thrombolysis, the vascular recanalization was effective, the neurological dysfunction was significantly improved, and the NIHSS score was reduced by more than 6 points was considered to be markedly effective. After 24 h of thrombolysis, the vascular recanalization was effective, neurological dysfunction was improved, with the ability of independent living and finishing work, but slow action, and the NIHSS score decreased more than 4 points were considered to be effective. After 24 h of thrombolysis, vascular stenosis occurred again, and the NIHSS score decreased less than 3 points were considered ineffective. Cure rate = (markedly effective + effective)/total × 100%.

*Vascular recanalization*: At 7 d after the operation, TICI was used for detection. The vessels occluded and without forward flow at the distal end was determined to be level 0. The contrast agent which partly passed through the occlusive site but could not fill the distal vessels was determined to be level 1. Contrast agent filling less than 2/3 of the ischemic zone of the affected vessels was determined as level 2a. The contrast agent which could fully fill the distal end of the artery with low speed of filling and emptying was determined to be level 2b. The contrast agent which could rapidly and completely fill the distal vessels and could be rapidly emptied was determined as level 3. Vascular recanalization rate = (level 3 + level 2)/total × 100%.

RETRACTED

*Adverse reaction*: Adverse reactions and complications from treatment to rehabilitation and hospitalization were recorded, and the incidence of adverse reactions was calculated.

*Hemodynamics*: Transcranial Doppler ultrasonography was used to detect bilateral cerebral artery blood flow before and at 10 d after treatment. The transducer frequency was set at 2.0 MHz; the maximum peak velocity (Vs), average velocity (Vm), vascular resistance index (RI), and pulsatility index (PI) were recorded.

*Nerve injury indexes*: levels of Glu, NES, and S100*β* in the serum of patients before and after treatment were detected.

*Clinical indexes*: Duration of coma and length of hospital stay of patients in the two groups were calculated.

*Prognosis*: After discharge, the patients were followed up for 3 months, which was conducted in the form of hospital review and investigated by the Glasgow Outcome Scale. Patients who returned to normal life but/or there were still some physiological disorders were judged to be good recovery. Patients who could live independently and conduct a certain degree of work and exercise under the protection were judged as a moderate disability. Patients who were unable to live independently and needed human care were judged as severe disability. Patients who were in a long-term persistent vegetative state but had a sleep cycle and eye activity were judged to be vegetative state. Patients who died during follow-up were judged as death.

### 3.4. Statistical Methods

All statistical analysis of the experimental results was performed by SPSS24.0 statistical software. All graph results were plotted by GraphPad 8. Enumeration data were expressed in the form of *n* (%), and the chi-square test was used for intergroup comparison. Measurement data were expressed in the form of mean ± standard deviation, and *t* test was used for intergroup comparison. *P* < 0.05 was considered statistically significant.

## 4. Results

### 4.1. Comparison of General Data

There were no significant differences in age, weight, BMI, onset time, gender, place of residence, infarction site, and complicated diseases between the two groups (*P* > 0.05), as shown in Table 1.

### 4.2. Comparison of NIHSS Score

There was no difference in the NIHSS score between the two groups before treatment (*P* > 0.05); after treatment, the NIHSS score was lower than that before the treatment (*P* < 0.05), while the NIHSS score in the group B was lower than that in the group A (*P* < 0.05), as shown in Figure 1.

RETRACTED

### 4.3. Comparison of Clinical Efficacy

The comparison of clinical efficacy between the two groups showed that the cure rate of group A was 81.16%, which was lower than that of group B (93.24%, *P* = 0.03), as shown in Table 2.

### 4.4. Comparison of Vascular Recanalization

The vascular recanalization of the two groups was compared, and it was found that there was no statistically significant difference between group A (78.26%) and group B (89.19%) (*P* > 0.05), as shown in Table 3.

### 4.5. Comparison of Adverse Reactions

The comparison of adverse reactions between the two groups showed that the incidence of adverse reactions in the group A was 18.84%, which was higher than that in the group B (6.76%), and the difference of incidence of adverse reactions between the two groups was statistically significant (*P* = 0.03), as shown in Table 4.

### 4.6. Comparison of Hemodynamics

The comparison of hemodynamics between the two groups showed that there was no difference in Vs, Vm, RI, and PI between the two groups before treatment (*P* > 0.05). After treatment, however, Vs and Vm increased, and RI and PI decreased (*P* < 0.05). After treatment, Vs and Vm in group A were lower than those in group B, and RI and PI were higher than those in group B (*P* < 0.05), as shown in Figure 2.

### 4.7. Comparison of Nerve Injury Indexes

The comparison of nerve injury indexes between the two groups showed that there was no difference in Glu, NES, and S100*β* between the two groups before treatment (*P* > 0.05). All of them decreased after treatment (*P* < 0.05). After treatment, Glu, NES, and S100*β* of group A were all higher than those of group B (*P* < 0.05), as shown in Figure 3.

### 4.8. Comparison of Clinical Indexes

By comparing the clinical indexes of the two groups, it was found that there was no significant difference in the duration of coma between the two groups (*P* > 0.05), while the length of hospital stay in group A was longer than that in group B (*P* > 0.05), as shown in Figure 4.

### 4.9. Comparison of Prognosis

The comparison of the prognosis of the two groups showed that there was no difference in the prognosis between the two groups (*P* > 0.05), as shown in Table 5.

## 5. Discussion

ACI, as a disease with a high incidence in the current middle-aged and elderly population, has not only a rapid onset but also a poor prognosis [14]. ACI is usually caused by cerebral atherosclerosis, which can lead to acute ischemia and hypoxia in the brain tissue. At this time, brain tissue is prone to necrosis, and brain death may occur once the optimal rescue opportunity is missed [15, 16]. Thrombolytic therapy is a commonly used method for the treatment of ACI, and the optimal treatment scheme is still controversial. It is extremely difficult to completely cure cerebral vascular diseases due to brain tissue necrosis, which is likely to cause lifelong neurological dysfunction diseases to patients [17, 18]. Therefore, by comparing the clinical efficacy of intra-arterial thrombolysis and arteriovenous thrombolysis combined with mechanical thrombectomy on ACI, and further analyzing the nerve injury of patients, this experiment is of great significance to the future clinical treatment of ACI patients for thrombolysis.

RETRACTED

The main cause of ACI is the formation of intravascular thrombosis, which obstructs the patency of blood circulation, and the purpose of thrombolytic therapy is to restore the patency of blood circulation by removing thrombolysis [19]. In clinical practice, intravenous thrombolysis is the initial thrombolytic therapy, which is performed by injecting thrombolytic drugs into the peripheral veins, circulating in the body, and reaching the thrombus for thrombolysis [20]. However, with the application of intravenous thrombolysis, scholars have found that the concentration of thrombolytic drugs would be greatly reduced after systemic circulation, and their thrombolytic effect is also seriously affected, and their therapeutic effect is increasingly insufficient [21]. Therefore, intra-arterial thrombolysis began to be widely used. Compared with intravenous thrombolysis, intra-arterial thrombolysis has a significant effect and a faster effect by injecting drugs directly into the body, but it has a certain limitation on the scope of action [22]. Combined with the advantages of the above two methods, arteriovenous thrombolysis can not only improve the efficiency of drug usage but also reduce the limitations of the scope of usage, which has been proved to have better efficacy than the single thrombolysis method [23]. With the application of minimally invasive technology in recent years, mechanical thrombectomy has gradually been widely used in clinical practice. Compared with traditional thrombolytic therapy, thrombectomy not only has a significant effect but also notably improves the recurrence and prognosis at the same time [24]. This experiment confirmed that the group B patients who received treatment of arteriovenous thrombolysis combined with mechanical thrombectomy had better clinical efficacy than the group A patients who received treatment of arteriovenous thrombolysis, suggesting that arteriovenous thrombolysis combined with mechanical thrombectomy had a more significant therapeutic effect on ACI patients. Lu et al. [25] were also relatively consistent with our research results, which can also support our experiment. In addition, we found that the NIHSS scores of Glu, NES, and S100*β* in group A were higher than those in group B after treatment, which also indicated that the use of arteriovenous thrombolysis and mechanical thrombectomy had less damage to the neurological function of patients. We speculated that the reason for the difference may be that although mechanical thrombectomy has a significant therapeutic effect, it has no improvement effect on the infarction of vascular endings. And in the process of thrombectomy, large and hard thrombus are difficult to combine with the stent. Moreover, mechanical stents may lead to thrombus fragmentation, and small blood clots that circulate with the bloodstream to the distal vessels may cause distal small vessel infarction [26]. At this time, arteriovenous thrombolysis can improve the results of thrombus elimination in patients, and on the other hand, broken and small thrombus can be eliminated through venous microcirculation, avoiding the recurrence of stenosis and improving the effect of recanalization of vessels. The comparison of adverse reactions between the two groups also showed that the incidence of adverse reactions in group A was higher than that in group B. The reason may be consistent with our conjecture. In addition, we compared the recanalization of blood vessels between the two groups of patients, and no significant difference was found between the two groups of patients, which also confirmed that both the two thrombolytic treatment regimens improved the vascular obstruction significantly, and was also in line with previous studies [27, 28]. However, by comparing the hemodynamic status of the two groups of patients, it could be seen that the hemodynamic status of the patients in group B was better than that in group A, indicating that arteriovenous thrombolysis and mechanical thrombectomy can improve the patients' intravascular environment more significantly. There was no difference in the duration of coma between the two groups, and the shorter hospital stay in group B compared with group A indicated that arteriovenous thrombolysis and mechanical thrombectomy could improve the rehabilitation cycle of patients, reducing the financial burden of treating ACI in the future. However, we compared the prognosis of patients in the two groups and found that there was no significant difference between the two groups, which we speculated might be caused by the small sample size included in this study. By observing the actual number of patients in the two groups who recovered well, we can see that there are more patients in group B than group A. Hence, we will expand the sample size as soon as possible and conduct a statistical analysis to improve our results.

RETRACTED

In this study, the clinical efficacy of arteriovenous thrombolysis and arteriovenous thrombolysis combined with mechanical thrombectomy on ACI was compared. Due to the limited experimental conditions, however, there are still shortcomings. Since the number of included subjects is small, the statistical calculation of partial results may be accidental. And because of the short experimental period, we could not evaluate the long-term prognosis of the two groups of patients. In addition, this experiment only compared the effect of thrombolytic therapy on ACI, without comparing the patients receiving conservative treatment. It was not clear whether there was any difference between the two in the comparison of various test results. We will conduct a more complete and comprehensive analysis on the above deficiencies as soon as possible to obtain better experimental results for clinical reference.

In conclusion, arteriovenous thrombolysis combined with mechanical thrombectomy has a significant effect on ACI, with high safety and quick effect. In addition, it has a stronger effect on improving and protecting the neurological function of patients, which is worth promoting in clinical practice.

## Figures and Tables

**Figure 1:** Comparison of NIHSS score in the two groups before and after treatment. ^∗^ represents the comparison of NIHSS score before treatment with that of the same group, *P* < 0.05. # represents the comparison of NIHSS score with group A after treatment, *P* < 0.05.

**Figure 2:** Comparison of hemodynamics. (a) Comparison of Vs between the two groups before and after treatment. (b) Comparison of Vm between the two groups before and after treatment. (c) Comparison of RI between the two groups before and after treatment. (d) Comparison of PI between the two groups before and after treatment. ^∗^ represents the comparison with that of the same group before treatment, *P* < 0.05. # represents the comparison with group A after treatment, *P* < 0.05.

**Figure 3:** Comparison of nerve injury indexes. (a) Comparison of Glu between the two groups before and after treatment. (b) Comparison of S100*β* between the two groups before and after treatment. (c) Comparison of NES between the two groups before and after treatment. ^∗^ represents the comparison with that of the same group before treatment, *P* < 0.05. # represents the comparison with group A after treatment, *P* < 0.05.

**Figure 4:** Comparison of clinical indexes between the two groups. (a) Comparison of duration of coma between the two groups. (b) Comparison of length of hospital stay. ^∗^ represents the comparison with group A, *P* < 0.05.

RETRACTED

**Table 1:** Comparison of general data (*n* (%)).

	Group A (*n* = 69)	Group B (*n* = 74)	*t* or *χ*^2^	*P*
Age (years)			1.204	0.231
	58.62 ± 6.92	57.16 ± 7.54		
BMI (kg/m^2^)			1.823	0.070
	26.62 ± 2.97	25.62 ± 3.54		
Onset time (h)			0.447	0.656
	5.62 ± 1.62	5.75 ± 1.84		
Gender				
Male	42 (60.87)	48 (64.86)		
Female	27 (39.13)	26 (35.14)		
Place of residence			0.244	0.621
City	42 (60.87)	48 (64.86)		
Countryside	27 (39.13)	26 (35.14)		
Infraction site			0.610	0.962
Basal ganglia	27 (39.13)	31 (41.89)		
Lobe	16 (23.19)	15 (20.27)		
Thalamus	12 (17.39)	15 (20.27)		
Cerebellum	10 (14.49)	10 (13.51)		
Brainstem	4 (5.80)	3 (4.05)		
Complicated disease			0.070	0.966
Coronary heart disease	36 (52.17)	40 (54.05)		
Hypertension	19 (27.54)	19 (25.68)		
Diabetes	14 (20.29)	15 (20.27)		

**Table 2:** Comparison of clinical efficacy between the two groups (*n* (%)).

	Group A (*n* = 69)	Group B (*n* = 74)	*χ* ^2^	*P*
Markedly effective	42 (68.87)	59 (79.73)	6.123	0.013
Effective	14 (20.29)	10 (13.51)	1.174	0.279
Ineffective	13 (18.84)	5 (6.76)	4.739	0.030
Cure rate (%)	81.16	93.24	4.739	0.030

**Table 3:** Comparison of clinical efficacy between the two groups (*n* (%)).

	Group A (*n* = 69)	Group B (*n* = 74)	*χ* ^2^	*P*
Level 0	8 (11.59)	5 (6.76)		
Level 1	7 (10.14)	3 (4.05)		
Level 2a	10 (14.49)	9 (12.16)		
Level 2b	19 (27.54)	25 (33.78)		
Level 3	25 (36.23)	32 (43.24)		
Recanalization rate (%)	78.26	89.19	3.159	0.076

**Table 4:** Comparison of adverse reactions between the two groups (*n* (%)).

	Group A (*n* = 69)	Group B (*n* = 74)	*χ* ^2^	*P*
Intracranial hemorrhage	2 (2.90)	1 (1.35)		
Gastrointestinal hemorrhage	2 (2.90)	1 (1.35)		
Urinary system hemorrhage	3 (4.35)	0 (0.00)		
Reperfusion injury	2 (2.90)	1 (1.35)		
Vascular reocclusion	4 (5.80)	2 (2.70)		
Incidence rate (%)	18.84	6.76	4.739	0.030

**Table 5:** Comparison of clinical efficacy between the two groups (*n* (%)).

	Group A (*n* = 69)	Group B (*n* = 74)	*χ* ^2^	*P*
Good recovery	34 (49.28)	46 (62.16)	2.406	0.121
Moderate disability	20 (28.99)	14 (18.92)	1.997	0.158
Severe disability	10 (14.49)	7 (9.46)	0.864	0.353
Persistent vegetative state	2 (2.90)	3 (4.05)	0.141	0.707
Death	4 (5.80)	4 (5.41)	0.010	0.919

## Data Availability

All the relevant data can be provided if any qualified researchers require.
